# Changes and Influencing Factors of Stress Disorder in Patients with Mild Traumatic Brain Injury Stress Disorder

This article has been retracted.

**DOI:** 10.1155/2022/9082946

**Published:** 2022-09-26

**Authors:** Chunmiao Xu, Qiang Li, Yin Gao, Hongliang Huo, Weixin Zhang

**Affiliations:** ^1^Nursing School, Qiqihar Medical University, Qiqihar, 161006 Heilongjiang, China; ^2^Department of Nursing, The Fourth Affiliated Hospital of Qiqihar Medical University, Qiqihar, 161000 Heilongjiang, China

## Abstract

Traumatic brain injury (TBI) is a brain injury caused by motor vehicle accidents, falls from heights, sports, and combat. Posttraumatic stress disorder (PTSD) is a complex mental disorder caused by physical and psychological trauma, which manifests itself with symptoms such as anxiety, depression, and cognitive dysfunction. How its symptoms arise and what factors influence it are not fully understood nor can it be predicted. In order to better understand the changes after stress disorder in TBI patients and the influencing factors of PTSD, this paper analyzed the changes and influencing factors of stress disorder in patients with mild traumatic brain injury stress disorder. In this paper, the Wechsler Memory Scale and functional magnetic resonance imaging were first used to study the memory impairment and functional changes of corresponding brain regions in patients with TBI stress disorder, and then, the Pittsburgh Sleep Quality Index Scale and the pain Visual Analogue Scale were used to study the influencing factors of PTSD. The results of the study showed that PTSD patients reduced and enhanced regional brain functional activity and impaired memory function in the resting state. Male gender, age under 45 years, no hemiplegia, and good sleep quality were protective factors for PTSD in TBI patients. The need for drug-assisted sleep, severe headache, and moderate headache was the risk factor for PTSD in TBI patients.

## 1. Introduction

Posttraumatic stress disorder become one of the most common psychiatric disorders, and different types of trauma cause it to vary in degree, which is considered as one of the top ten mental illnesses that seriously damage people's health. The rapid development of medical imaging technology in the past two decades, especially the development of functional magnetic resonance imaging technology, has made it possible to study the brain structure and function of patients with PTSD in vivo, which has opened up a new perspective for the diagnosis of PTSD. Research on the influencing factors of PTSD can enable early identification and timely intervention of patients, which can significantly reduce the incidence of PTSD. Therefore, this paper analyzed the changes and influencing factors of stress disorder in patients with mild traumatic brain injury stress disorder.

Many scholars have studied the changes of patients with posttraumatic stress disorder. Monsour et al. described the underlying pathophysiology of TBI and PTSD symptoms and investigated stem cell treatment options [1]. Mallol-Ragolta and Dhamija proposed a multimodal approach to predict changes in PTSD symptom severity [2]. Vermetten and Germain studied the relationship between posttraumatic stress disorder and sleep changes in patients [3]. Segal and Wald used data from a group of male infantry soldiers to study changes in the PTSD symptom network from precombat to postcombat [4]. Atmaca et al. studied the pituitary volume in PTSD patients and found that the pituitary volume of PTSD patients was smaller than that of other healthy control patients [5]. Although there are many studies on the changes of PTSD patients, the PTSD changes in TBI patients still need further research.

At present, there are many studies on the influencing factors of PTSD. Reijnen studied the risk factors affecting the occurrence of PTSD [6]. Bramblett examined gender relations and symptom presentation in patients with PTSD [7]. Smock identified risk factors for posttraumatic stress disorder in people who experienced a disaster [8]. Wilkerson analyzed the impact of smell and the central olfactory system in the pathophysiology of PTSD [9]. Lewis explored the relationship between PTSD and genetic variation in widely theorized molecular targets [10]. Although there are many studies on the influencing factors of PTSD, there are fewer studies on the influencing factors of PTSD in TBI patients, which provided scientific basis for psychological intervention strategies and measures for TBI patients.

In this paper, the Wechsler Memory Scale and functional magnetic resonance imaging were first used to analyze the memory changes and changes in brain functional activity after PTSD in TBI patients, and then, the Pittsburgh Sleep Quality Index Scale and the pain Visual Analogue Scale were used to study the influencing factors of PTSD in TBI patients.

## 2. Memory Impairment and Functional Changes of Corresponding Brain Regions in Patients with TBI Stress Disorder

### 2.1. Experimental Subjects

TBI patients who are treated in the Second Affiliated Hospital of Qiqihar Medical from January 2020 to December 2021 are selected as the research subjects, including 10 patients with PTSD and 10 patients without PTSD. The PTSD patients are named the PTSD group, and the patients without PTSD are named the non-PTSD group [11].

### 2.2. Experimental Tools

#### 2.2.1. Wechsler Memory Scale (WMS)

WMS is an objective memory test method commonly used in clinical practice, which helps to identify organic and functional memory impairment. The table is divided into two types: A and B. The scale consists of seven subtests, namely, common sense, orientation, numerical sequence relationship, logical memory, numerical breadth, visual memory, and paired word associative learning, which combine scores from the seven items to yield a memory quotient (MQ), and the MQ for the normal level of the WMS is 100 [12].

#### 2.2.2. Functional Magnetic Resonance Imaging (fMRI)

fMRI is now used to study the intrinsic functional organization of the brain, and blood oxygen level dependence (BOLD) is used to investigate the activation of the resting state of the brain. fMRI is used to study the brain responses to intrinsically synchronized coordination in the resting state. Often by detecting the regional homogeneity (ReHo) of the BOLD signal, the Kendall concordance coefficient (KCC) is used to represent the local consistency of the selected voxel and the adjacent voxels in the same time series, and the KCC value is assigned to this voxel, and the value range is 0-1 [13]. The functional magnetic resonance imaging calculation method is shown in Figure 1.

In a normal workflow, after fMRI data is collected, it is transferred from the scanner to a server and then analyzed offline over weeks, months, or years. It is analyzed during data collection rather than after data collection [14].

ReHo measures the consistency of the temporal signal between a voxel and surrounding voxels, which is a parameter calculated based on the Kendal harmony coefficient [15]. It is assumed that the order of the signal value *i* collected by a body at time *j* in the entire time series is *rn*, and the total ranking *R* of all studied voxels at time *i* is

(1) $$\begin{array}{c} R_{i}=\overset{K}{\underset{j=1}{\sum }}r_{i,j}, \end{array}$$

where *K* is the number of study local voxels, generally 27.

The average of *R* over all times is

(2) $$\begin{array}{c} \bar{R}=\frac{1}{N}\overset{N}{\underset{i=1}{\sum }}R_{i}. \end{array}$$

Then, ReHo can be calculated based on the following formula:

(3) $$\begin{array}{c} \text{ReHo}=\frac{12\sum_{i=1}^{N}{\left(R_{i}-\bar{R}\right)}^{2}}{K^{2}\left(N^{3}-N\right)}. \end{array}$$

The higher the ReHo value, the better the consistency between local voxels and neighboring voxels.

In this paper, the ReHo method was used to investigate the changes of brain function in PTSD patients in the resting state.

### 2.3. Data and Statistical Analysis

The PTSD Checklist-Civilian version (PCL-C) scale and the WMS are collected from the study patients, the questionnaires are filled out by themselves without external interference during the investigation process, and the patients are subjected to fMRI testing two weeks after TBI with consent [16].

In the ReHo analysis part, based on the ReHo hypothesis, the Kendall harmony coefficient is used to measure the time series similarity in the local brain area. In this paper, each of the adjacent 27 voxels is defined as a voxel group, the KCC value is assigned to the central voxel of this cube voxel group, and the calculation formula is as follows:

(4) $$\begin{array}{c} W=\frac{\sum {\left(R_{i}\right)}^{2}-n{\left(\bar{R}\right)}^{2}}{\left(1/12\right)K^{2}\left(n^{2}-n\right)}, \end{array}$$

where *W* is the total KCC value of the selected voxels, and the value range is 0-1; *R*_*i*_ is the rank sum of the *i*-th time point; $\bar{R}$ is the average value; *K* is the number of time series (*K* = 27); and *n* is the total rank (here *n* = 235 time points).

The ReHo image of each subject is calculated by the REST software to obtain the normalized KCC value of each voxel, and then, the voxels at the corresponding positions in the two sets of KCC images obtained by the ReHo method are tested and analyzed. The abnormal brain regions obtained are regarded as regions of interest (ROI), and the average ReHo value in each subject's ROI is extracted. The obtained data are analyzed by the SPSS19.0 statistical software, and *P* < 0.05 two-sided test indicates that the test is statistically significant meaning [17].

## 3. Evaluation of Influencing Factors of Stress Disorder in TBI Patients

### 3.1. Experimental Subjects

A total of 100 TBI patients who are treated in the Second Affiliated Hospital of Qiqihar Medical from January 2020 to December 2021 are selected as the research objects.

### 3.2. Experimental Tools

The inpatients who meet the inclusion criteria are surveyed by trained investigators after they enter a stable recovery period, and PTSD is diagnosed by a psychiatrist. The contents of the questionnaire include general situation questionnaire, Pittsburgh Sleep Quality Index Scale (PSQI), and pain Visual Analog Scale (VAS) [18].

#### 3.2.1. Pittsburgh Sleep Quality Index Scale

The PSQI consists of 18 self-assessed items, including 7 components, sleep quality, sleep onset time, sleep duration, sleep efficiency, sleep disturbance, hypnotic drugs, and daytime dysfunction. The item score ranges from 0 to 3 points, and the total score ranges from 0 to 21 points. The higher the score, the worse the sleep quality. When the PSQI total score ≥ 7 points, the individual is considered to have sleep disorders; when the PSQI total score is less than 5 points, the sleep quality is considered to be good; when the score is between the two, the sleep quality is considered to be average. A single dimension score > 1 point indicates that there is a sleep problem in this dimension [19].

#### 3.2.2. Pain Visual Analog Scale

VAS is a 10 cm long scale, with 0 at one end of the scale representing “no pain” and 10 at the other end representing “severe pain.” The patient locates the degree of pain on a straight line according to his/her self-feeling. A score of 1-3.3 indicates mild pain, and a score of 3.3-6.6 indicates moderate pain, and a score of 6.6-10 indicates severe pain [20], as shown in Figure 2.

## 4. Experimental Results of Memory Impairment and Functional Changes of Corresponding Brain Regions in Patients

### 4.1. WMS Measurement Results

The first WMS test is carried out two weeks after the occurrence of TBI, and the second WMS test is carried out 3 months after the occurrence of TBI. The test results are expressed in the form of mean ± standard deviation: ∗ means *P* < 0.05, and ∗∗ means *P* < 0.01.

#### 4.1.1. Common Sense Test

The common sense test results are shown in Table 1 and Figure 3.

As can be seen from the data, when the common sense test is conducted for the first time, the mean test result of the PTSD group is 7.32, and the mean test result of the non-PTSD group is 9.85. In the second general knowledge test, the mean of the test results in the PTSD group increases to 8.66, and the mean of the test results in the non-PTSD group increases to 10.49. The ability of common sense memory in both groups is greatly improved, and the data in the PTSD group at the second measurement is *P* < 0.01, which indicates that the difference in common sense of the patients 3 months after the trauma is statistically significant.

#### 4.1.2. Orientation Test

The orientation test results are shown in Table 2 and Figure 4.

On the first orientation test, the mean test result in the PTSD group is 8.58. On the second orientation test, the mean test result in the PTSD group decreases to 7.32. In the non-PTSD group, the mean of the first measurement is 11.26, and the mean of the second measurement increases to 11.85. The directional memory ability of non-PTSD patients is improved, and the data in the PTSD group at the second test is *P* < 0.01, which indicates that the differences in the orientation of the patients 3 months after the trauma are statistically significant.

#### 4.1.3. Number Sequence Relationship Test

The numerical sequence test results are shown in Table 3 and Figure 5.

The mean test result of the PTSD group at the first test in the numerical order relation is 9.24, and the mean test result of the non-PTSD group is 12.57. In the numerical sequence relationship, the mean test result of the PTSD group at the second test is 8.73, and the mean test result of the non-PTSD group is 14.69. Comparing the results of the two tests, it can be seen that the results of the second test in the PTSD group are lower than those in the first test, and the results of the second test in the non-PTSD group are significantly improved compared with the first test. In the second test, the data of the PTSD group and the non-PTSD group are *P* < 0.05, which indicate that the difference in the numerical order of the patients 3 months after the trauma is statistically significant.

#### 4.1.4. Logical Memory Test

The logical memory test results are shown in Table 4 and Figure 6.

In the first test of logical memory, the mean test result in the PTSD group is 7.26, and the mean test result in the non-PTSD group is 10.56. In the second test of logical memory, the mean test result of the PTSD group is 7.83, and the mean test result of the non-PTSD group is 12.78. Comparing the results of the two tests, it can be seen that the results of the second test in the PTSD group are improved compared with the first test, and the results of the second test in the non-PTSD group are significantly improved compared with the first test. The data of the PTSD group at the first test and the second test are *P* < 0.01, indicating that the differences in logical memory of trauma patients are statistically significant.

#### 4.1.5. Digital Breadth Test

The digital breadth test results are shown in Table 5 and Figure 7.

The mean test result for the PTSD group on the first test of digital span is 6.92, and the mean test result for the non-PTSD group is 8.75. The mean of the test results of the PTSD group is 5.48 in the second test, and the mean of the test results of the non-PTSD group is 11.36. Comparing the results of the two tests, it can be seen that the results of the second test in the PTSD group are lower than those in the first test, and the results of the second test in the non-PTSD group are significantly improved compared with the first test. The data of the PTSD group in the second test is *P* < 0.05, indicating that the difference in the number of patients is statistically significant 3 months after the trauma.

#### 4.1.6. Visual Memory Test

The visual memory test results are shown in Table 6 and Figure 8.

In the first test of visual memory, the mean test result in the PTSD group is 7.69, and the mean test result in the non-PTSD group is 10.68. On the second test of visual memory, the mean test result in the PTSD group is 8.13, and the mean test result in the non-PTSD group is 11.56. Comparing the results of the two tests, it can be seen that the results of the second test in the PTSD group and the non-PTSD group are improved compared with the first test.

#### 4.1.7. Paired Word Association Learning Test

The test results of paired word association learning are shown in Table 7 and Figure 9.

In the first test of paired word association learning, the mean test result of the PTSD group is 6.51, and the mean of the test result of the non-PTSD group is 9.36. In the second test of paired word association learning, the mean test result of the PTSD group is 5.49, and the mean of the test result of the non-PTSD group is 10.87. Comparing the results of the two tests, it can be seen that the results of the second test in the PTSD group are lower than those in the first test, and the results of the second test in the non-PTSD group are improved compared with the first test. The data of the PTSD group in the second test is *P* < 0.05, indicating that the difference in paired word association learning is statistically significant 3 months after the trauma.

WMS is assessed in all subjects two weeks after the trauma, and it is found that there is a statistically significant difference in logical memory between the PTSD group and the non-PTSD group, indicating that PTSD patient experience memory impairment in the early stages of traumatic events, and it is mainly manifested as a certain degree of damage to short-term memory, instantaneous memory, and visual memory. Measurements of WMS 3 months after the traumatic event find statistically significant differences between the two groups in common sense, orientation, number sequence, logical memory, number span, and paired word associative learning. It can be inferred that PTSD patients may be impaired in auditory-verbal memory, short-term memory, and instantaneous memory compared with non-PTSD patients. After experiencing traumatic events, patients would have some memory impairment in the early stage, and the memory function of the non-PTSD population would gradually recover over time.

### 4.2. Comparison of ReHo Values of Patients

#### 4.2.1. Comparison of ReHo Values between the Two Groups of TBI Patients Two Weeks after Trauma

The ReHo values of the two groups of TBI patients are compared two weeks after the trauma, and the brain regions with ReHo values that differed between the PTSD group and the non-PTSD group are shown in Table 8.

It can be seen from the data that two weeks after the trauma, the brain region with the largest difference in ReHo value between the PTSD group and the non-PTSD group is the right occipital lobe/lingual gyrus. The number of voxels in the region is 24, and the *t* value is -7.28.

#### 4.2.2. Comparison of ReHo Values between the Two Groups of TBI Patients 3 Months after Trauma

The ReHo values of the two groups of TBI patients are compared 3 months after the trauma, and the brain regions with ReHo values differing between the PTSD group and the non-PTSD group are shown in Table 9.

It can be seen from the data that 3 months after the trauma, the brain regions with lower ReHo values in the PTSD group than those in the non-PTSD group are the right middle temporal gyrus, right occipital lobe, left inferior temporal gyrus, and right precentral gyrus. The brain regions with higher ReHo values in the PTSD group than in the non-PTSD group are the left cerebellum, left inferior frontal gyrus, left superior temporal gyrus, left thalamus, right middle occipital gyrus, right middle cingulate gyrus, right paracentral gyrus lobe, and right upper frontal gyrus. Among them, the number of voxels in the right middle temporal gyrus is 5, and the *t* value is -4.92; the number of voxels in the right occipital lobe is 1, and the number of voxels in the *t* value is -416; the number of voxels in the left inferior temporal gyrus is 3, and the *t* value is -6.05; the number of voxels in the right precentral gyrus is 2, and the *t* value is 4.32; the number of voxels in the left cerebellar gyrus is 4, and the number of *t* values is 5.46; the number of voxels in the left inferior frontal gyrus is 2, and the *t* value is -4.57; the number of voxels in the left superior temporal gyrus is 1, and the *t* value is -4.86; the number of voxels in the left thalamus is 9, and the *t* value is 7.39; the number of voxels in the right middle occipital gyrus is 1, and the *t* value is -5.83; the number of voxels in the right middle cingulate gyrus is 2, and the *t* value is 4.57; the number of voxels in the right paracentral lobule is 3, and the *t* value is 4.79; the number of voxels in the right superior frontal gyrus is 3, and the *t* value is 5.32.

#### 4.2.3. Comparison of ReHo Values before and after PTSD Group

The ReHo value at two weeks and the ReHo value at 3 months in the PTSD group are compared, and the results are shown in Table 10.

It can be seen from the data that the brain regions with the ReHo value at 3 months lower than the ReHo value at 2 weeks in the PTSD group are the left cingulate gyrus, the right precuneus, and the left superior parietal lobe. In the PTSD group, the brain regions whose ReHo value at 3 months is higher than that at 2 weeks are the right orbital gyrus, right inferior frontal gyrus, and left superior frontal gyrus. Among them, the number of voxels in the left cingulate gyrus is 1, and the *t* value is 5.64; the number of voxels in the right precuneus is 2, and the value of *t* is -5.73; the number of voxels in the left upper parietal lobe is 1, and the value of *t* is -3.86; the number of voxels in the orbital gyrus of the right frontal lobe is 2, and the *t* value is 4.98; the number of voxels in the right inferior frontal gyrus is 1, and the *t* value is 6.07; the number of voxels in the left superior frontal gyrus is 2, and the *t* value is 5.69.

#### 4.2.4. Comparison of ReHo Values before and after Non-PTSD Group

The ReHo value at 2 weeks and the ReHo value at 3 months in the non-PTSD group are compared, and the results are shown in Table 11.

It can be seen from the data that the left occipital lobe is the brain region with the largest difference in ReHo value between two weeks after trauma and 3 months after trauma in the non-PTSD group. The ReHo value of this brain area at 3 months is higher than that at 2 weeks. The number of voxels in the brain area is 2, and the *t* value is 5.14.

Abnormal neural activity in these brain regions may be involved in the development and persistence of symptoms in patients with PTSD. The middle temporal gyrus inhibits amygdala function, promotes extinction of fear conditioning, and is associated with episodic memory and higher-order language processing. The decrease in the regional consistency of this brain region makes it difficult for PTSD patients to fade fear memory and the function of verbal memory decline, and symptoms such as flashback, amnesia, and increased alertness occur. The occipital lobe is the center of basic visual processing. The results of the study show that the ReHo value of the right occipital lobe decreases and the ReHo value of the right middle occipital gyrus increases. The abnormal function of the occipital lobe may be related to the flashback symptoms of traumatic events, and the thalamus is related to memory, consciousness regulation, sleep, and language, which is involved in regulating the interaction of attention and vigilance. The results of the study show that the ReHo value of the left thalamus is increased, which reflects the hyperactivity of this area. This may be related to the hypervigilance state and sleep disturbance in patients after traumatic events.

## 5. Experimental Results of the Evaluation of the Influencing Factors of Stress Disorder in TBI Patients

### 5.1. Survey on the General Condition of Patients

The results of the general survey of the patients are shown in Table 12.

From the data, among the 100 TBI patients, 30 have moderate PTSD, 18 have moderate PTSD, and 52 have no PTSD. In the survey of four general factors of gender, age, marital status, and occupational nature, the *P* value of gender and age is less than 0.001, which is statistically significant.

### 5.2. Pittsburgh Sleep Quality Index Scale

#### 5.2.1. The Patient's Sleep Disorder Level

The average scores of 7 dimensions in the PSQI table and the total PSQI scores of the 100 TBI patients are shown in Table 13 and Figure 10.

In the test results of the 7 dimensions of the PSQI table, the average scores of TBI patients are higher than the domestic norm of PSQI. For sleep quality, the mean score of TBI patients is 1.16, and the mean domestic norm is 0.65. For sleep time, the mean score of TBI patients is 0.98, and the mean domestic norm is 0.52. For sleep time, the mean score of TBI patients is 1.76, and the mean domestic norm is 0.61. For sleep efficiency, the mean score of TBI patients is 0.35, and the mean domestic norm is 0.18. For sleep disorders, the mean score of TBI patients is 1.26, and the mean domestic norm is 0.73. For hypnotic drugs, the mean score of TBI patients is 1.58, and the mean domestic norm is 0.86. For daytime dysfunction, the mean score of TBI patients is 1.26, and the mean domestic norm is 0.43. The mean PSQI total score of TBI patients is 7.84, and the mean PSQI total score of domestic norm is 3.88. The *P* value of each data is less than 0.001, and the data difference is statistically significant.

#### 5.2.2. Difference Analysis of Sleep Disturbance among Different PTSD Symptom Groups

Differences in sleep disturbance among patients with severe PTSD, moderate PTSD, and no PTSD are shown in Table 14.

For the 3 groups of patients, the order of data size is severe PTSD > moderate PTSD > none PTSD. For sleep quality, patients with severe PTSD score a mean score of 1.93, patients with moderate PTSD score a mean score of 1.37, and patients without PTSD score a mean score of 0.75. For sleep time, the mean score is 1.58 in patients with severe PTSD, 0.96 in patients with moderate PTSD, and 0.47 in patients without PTSD. For sleep duration, the mean score for patients with severe PTSD is 2.13, the mean score for patients with moderate PTSD is 1.97, and the mean score for patients without PTSD is 1.62. For sleep efficiency, the mean score for patients with severe PTSD is 1.16, the mean score for patients with moderate PTSD is 0.74, and the mean score for patients without PTSD is 0.31. For sleep disturbance, the mean score is 1.37 for those with severe PTSD, 1.14 for those with moderate PTSD, and 0.85 for those without PTSD. For hypnotics, the mean score is 1.67 for patients with severe PTSD, 1.24 for those with moderate PTSD, and 0.95 for patients without PTSD. For daytime dysfunction, the mean score is 1.39 for those with severe PTSD, 1.05 for those with moderate PTSD, and 0.71 for those without PTSD. The mean PSQI total score of patients with severe PTSD is 10.63, the mean PSQI total score of patients with moderate PTSD is 8.58, and the mean PSQI total score of patients without PTSD is 5.37. The *P* value of each data is less than 0.005, and the data difference is statistically significant.

### 5.3. Multivariate Analysis of the Influencing Factors of PTSD in TBI Patients

Taking PTSD as the dependent variable, univariate analysis is performed on TBI patients to study the influencing factors of PTSD, and the results are shown in Table 15.

The experimental results of various factors are analyzed. The OR value of male patients is 0.286, and the 95% CI is between 0.273 and 0.569, *P* < 0.001, which indicate that male TBI patients have milder PTSD responses and gender can affect the degree of PTSD response in TBI patients. The OR value of age below 45 years is 0.117, and 95% CI is between 0.058 and 0.304, *P* < 0.001; for patients aged 45 to 60 years, the OR value is 0.562, the 95% CI is 0.495-1.378, and the *P* value is 0.146. It shows that age can affect the degree of PTSD response in TBI patients, and TBI patients under 45 years old have milder PTSD response. The OR value of severe headache patients is 4.793, and 95% CI is between 3.352 and 13.497; the OR value of moderate headache patients is 1.465, and 95% CI is between 0.287 and 1.153, which indicate that headache is an influencing factor for increasing PTSD response in TBI patients. The OR value of patients without hemiplegia is 0.389, the 95% CI is between 0.242 and 0.679, and the *P* value was 0.001. It shows that hemiplegia can increase the degree of PTSD response in TBI patients, and the PTSD response in patients without hemiplegia is milder. The OR value of patients with good sleep quality is 0.147, with a 95% CI between 0.067 and 0.354; the OR value of patients with good sleep is 0.388, with a 95% CI between 0.246 and 0.728; the OR value of patients with normal sleep is 0.649, and 95% CI is between 0.352 and 1.077. It shows that sleep quality affects the degree of PTSD response in TBI patients. The better the sleep quality, the lighter the PTSD response in TBI patients. The OR value of patients requiring drug-assisted sleep is 2.873, and the 95% CI is between 1.453 and 3.682, which indicate that drug-assisted sleep is a risk factor for PTSD in TBI patients.

In conclusion, male gender, age under 45 years, no hemiplegia, and good sleep quality can reduce the severity of PTSD in TBI patients. The need for medication to assist sleep, severe headache, and moderate headache exacerbates the severity of PTSD in TBI patients.

## 6. Conclusions

In this paper, WMS and fMRI were used to study the changes of memory function and functional activity of brain regions after PTSD in TBI patients. The results of the study showed that the auditory verbal memory, short-term memory, and instantaneous memory might be impaired in TBI patients after PTSD, and the neurogenesis in the brain area was abnormal. By using PQSI and VAS to study the influencing factors of PTSD in TBI patients, the results of the study showed that gender, age, hemiplegia, sleep, and headache all affected the severity of PTSD in patients. Patients were less likely to develop PTSD if they met the following conditions: male, under 45 years of age, no hemiplegia, and good sleep quality; patients were more likely to develop PTSD with the following conditions: need for medication to aid sleep, severe headache, and moderate headache.

## Figures and Tables

**Figure 1:** Functional magnetic resonance imaging computational methods.

**Figure 2:** Pain Visual Analog Scale.

**Figure 3:** WMS common sense measurement results.

**Figure 4:** WMS orientation measurement results.

**Figure 5:** WMS number order measurement results.

**Figure 6:** WMS logical memory measurement results.

**Figure 7:** WMS digital breadth measurement results.

**Figure 8:** WMS visual memory measurement results.

**Figure 9:** WMS paired word association measurement results.

**Figure 10:** Average score on 7 dimensions of PSQI table.

**Table 1:** WMS common sense measurement results.

Quiz item		Common sense
First measurement	PTSD group	7.32 ± 1.58
	Non-PTSD group	9.85 ± 0.94

Second measurement	PTSD group	8.66 ± 1.47^∗∗^
	Non-PTSD group	10.49 ± 0.85

**Table 2:** WMS orientation measurement results.

Quiz item		Orientation
First measurement	PTSD group	8.58 ± 2.13
	Non-PTSD group	11.26 ± 1.49

Second measurement	PTSD group	7.32 ± 1.97^∗∗^
	Non-PTSD group	11.85 ± 1.62

**Table 3:** WMS number order measurement results.

Quiz item		Number order
First measurement	PTSD group	9.24 ± 3.86
	Non-PTSD group	12.57 ± 2.42

Second measurement	PTSD group	8.73 ± 2.28^∗^
	Non-PTSD group	14.69 ± 1.92^∗^

**Table 4:** WMS logical memory measurement results.

Quiz item		Logical memory
First measurement	PTSD group	7.26 ± 1.43^∗∗^
	Non-PTSD group	10.56 ± 2.01

Second measurement	PTSD group	7.83 ± 1.95^∗∗^
	Non-PTSD group	12.78 ± 2.14

**Table 5:** WMS digital breadth measurement results.

Quiz item		Digital breadth
First measurement	PTSD group	6.92 ± 3.53
	Non-PTSD group	8.75 ± 1.69

Second measurement	PTSD group	5.48 ± 2.74^∗^
	Non-PTSD group	11.36 ± 1.28

**Table 6:** WMS visual memory measurement results.

Quiz item		Visual memory
First measurement	PTSD group	7.69 ± 2.44
	Non-PTSD group	10.68 ± 1.26

Second measurement	PTSD group	8.13 ± 2.07
	Non-PTSD group	11.56 ± 1.73

**Table 7:** WMS paired word association measurement results.

Quiz item		Paired word association
First measurement	PTSD group	6.51 ± 3.27
	Non-PTSD group	9.36 ± 1.24

Second measurement	PTSD group	5.49 ± 2.62^∗^
	Non-PTSD group	10.87 ± 1.65

**Table 8:** Brain regions with different ReHo values after two weeks.

Different brain regions		Right occipital/lingual gyrus
Number of voxels		24
*t* value of the point of maximum difference		-7.28

Maximum difference point MNI coordinate	*X*	19
	*Y*	-76
	*Z*	-4

**Table 9:** Brain regions with different ReHo values after 3 months.

Different brain regions		Number of voxels	*t* value of the point of maximum difference	Maximum difference point MNI coordinate		
				*X*	*Y*	*Z*
Lower brain regions than non-PTSD	Right middle temporal gyrus	5	-4.92	56	-12	-19
	Right occipital lobe	1	-416	27	-87	-17
	Left inferior temporal gyrus	3	-6.05	-45	-13	-26
	Right precentral gyrus	2	4.32	34	-28	49

Higher than non-PTSD brain regions	Left cerebellum	4	5.46	-51	-49	-46
	Left inferior frontal gyrus	2	-4.57	-49	26	-19
	Left superior temporal gyrus	1	-4.86	-63	10	-8
	Left thalamus	9	7.39	-18	-31	9
	Right middle occipital gyrus	1	-5.83	30	-92	34
	Right middle cingulate	2	4.57	14	-30	43
	Right paracentral lobule	3	4.79	5	--24	51
	Right upper forehead	3	5.32	19	37	66

**Table 10:** Comparison of ReHo values at 2 weeks and 3 months in the PTSD group.

Different brain regions		Number of voxels	*t* value of the point of maximum difference	Maximum difference point MNI coordinate		
				*X*	*Y*	*Z*
Brain regions less than 2 weeks old	Left cingulate	1	5.64	-5	-11	25
	Right precuneus	2	-5.73	24	-56	56
	Left upper parietal lobe	1	-3.86	-12	-59	56

Brain regions older than 2 weeks	Right frontal orbital gyrus	2	4.98	21	40	-27
	Right inferior frontal gyrus	1	6.07	50	23	-12
	Left upper forehead	2	5.69	-32	63	9

**Table 11:** Comparison of ReHo values at 2 weeks and 3 months in the non-PTSD group.

Different brain regions		Left occipital lobe
Number of voxels		2
*t* value of the point of maximum difference		5.14

Maximum difference point MNI coordinate	*X*	-40
	*Y*	-68
	*Z*	0

**Table 12:** Patient general survey results.

Factors		Severe PTSD	Moderate PTSD	None PTSD	Total	*χ* ^2^	*P* value
Gender	Female	16	8	22	46	17.952	<0.001
	Male	14	10	30	54		

Age	<45	13	4	15	32	34.578	<0.001
	45-60	7	6	18	31		
	>60	10	4	23	37		

Marital status	Widowed	8	3	8	19	0.461	0.638
	Unmarried	4	1	13	18		
	Married	25	7	31	63		

Occupational nature	Mental work	8	2	15	25	3.764	0.084
	Combination of brain and physical strength	18	3	32	53		
	Manual labor	8	4	10	22		

**Table 13:** Average score on 7 dimensions of PSQI table.

Project	The average score	The domestic norm	*t*	*P*
The quality of sleep	1.16 ± 0.41	0.65 ± 0.82	9.64	<0.001
Time to fall asleep	0.98 ± 0.67	0.52 ± 0.33	11.58	<0.001
Sleeping time	1.76 ± 0.81	0.61 ± 0.49	41.83	<0.001
Sleep efficiency	0.35 ± 0.72	0.18 ± 0.24	7.62	<0.001
Sleep disorder	1.26 ± 0.84	0.73 ± 0.38	9.47	<0.001
Hypnotic drugs	1.58 ± 0.74	0.86 ± 0.47	26.92	<0.001
Daytime dysfunction	1.26 ± 0.75	0.43 ± 0.52	5.46	<0.001
PSQI total score	7.84 ± 1.62	3.88 ± 2.52	32.83	<0.001

**Table 14:** Differences in sleep disturbance among different PTSD symptom groups.

Project	Severe PTSD	Moderate PTSD	None PTSD	*t*	*P*
The quality of sleep	1.93 ± 1.52	1.37 ± 0.54	0.75 ± 0.86	3.57	0.001
Time to fall asleep	1.58 ± 1.06	0.96 ± 1.24	0.47 ± 0.92	3.18	0.001
Sleeping time	2.13 ± 0.88	1.97 ± 1.04	1.62 ± 0.56	4.68	0.016
Sleep efficiency	1.16 ± 0.41	0.74 ± 0.66	0.31 ± 0.58	11.79	<0.001
Sleep disorder	1.37 ± 0.96	1.14 ± 0.28	0.85 ± 0.32	3.48	0.035
Hypnotic drugs	1.67 ± 1.02	1.24 ± 0.69	0.95 ± 0.27	4.96	<0.001
Daytime dysfunction	1.39 ± 0.76	1.05 ± 1.24	0.71 ± 0.48	3.06	0.009
PSQI total score	10.63 ± 1.85	8.58 ± 2.74	5.37 ± 0.82	13.87	<0.001

**Table 15:** Multivariate analysis of the influencing factors of PTSD in TBI patients.

Variable		Reference group	*P* value	OR value	95% CI of OR
Gender	Male	Female	<0.001	0.286	0.273-0.569

Age	<45	>60	<0.001	0.117	0.058-0.304
	45-60	—	0.146	0.562	0.495-1.378

Headache	Severe headache	Painless and mild	<0.001	4.793	3.352-13.497
	Moderate headache	—	0.032	1.465	0.287-1.153

Hemiplegia	No	Yes	0.001	0.389	0.242-0.679

Sleep quality	Very good	Very poor	<0.001	0.147	0.067-0.354
	Good	—	0.007	0.388	0.246-0.728
	Generally	—	0.067	0.649	0.352-1.077

Drug-assisted sleep	Yes	No	<0.001	2.873	1.453-3.682

## Data Availability

The data of this paper can be obtained through sending email to the authors.
